The article "The Study of Maslow's Hierarchy of Needs Theory in the Doctor-Nurse Integration Teaching Method on Clinical Interns" was retracted in 2023. Reasons: signs of a paper mill; suspected computer-generated content; unreliable results or conclusions; lack of ethics approval or compliance.

# The Study of Maslow's Hierarchy of Needs Theory in the Doctor-Nurse Integration Teaching Method on Clinical Interns

**DOI:** 10.1155/2022/6388068

**Published:** 2022-04-18

**Authors:** Zhe Liu, Junying Xiang, Fangjing Luo, Xiaoli Hu, Ping Luo

**Affiliations:** Department of Gastroenterology, Clinical Medical College and Affiliated Hospital of Chengdu University, Chengdu University, Chengdu 610081, China

## Abstract

The student's attitude towards the doctor-nurse integrated teaching model and Maslow's hierarchy of needs theory is an important topic in clinical teaching. In this study, choosing 134 intern doctors and practice nurses who intern from January to December 2020. 67 students are selected as the control group, and the traditional interns teaching mode is adopted. 67 students are selected as the experimental group and Maslow's hierarchy of needs theory to apply in the doctor-nurse integrated teaching mode. The results show that the doctor-nurse integrated teaching model are accepted by most students, and the application of Maslow's hierarchy of needs theory in the clinical interns has advantages over the traditional model.

## 1. Introduction

The American humanist psychologist Maslow first proposed the hierarchy of needs theory in 1954. This theory is structured to divide people's needs into five levels from low to high, namely, physiological needs, safety needs, love, and a sense of belonging, the needs of people, the needs of respect, and the needs of self-realization. Internship teaching is an important part of medical undergraduate teaching. Deepening the reform of internship teaching is the top priority of talent training and an important way to improve students' independent learning ability, innovation ability, clinical thinking ability, and job competence [1, 2]. In the internship teaching work of undergraduate medical and nursing interns, our department conducts evaluations according to their learning needs and key points and adopts the teaching methods of medical and nursing integration, so as to evaluate the application of Maslow's need-level theory in medical internship teaching and the integration of medical and nursing, evaluation of teaching development [3, 4].

The rest of this study is organized as follows: Section 2 discusses related work, followed by the case study methods and observational indicators in Section 3. The case analysis and comparison is discussed in Section 4.  Section 5 concludes the study with summary and future research directions.

## 2. Related Work

In recent years, the Ministry of Education has subsequently issued “Several Opinions on Comprehensively Improving the Quality of Higher Education,” “Several Opinions on Further Strengthening the Practice of Educating People in Colleges and Universities,” and “Guiding Opinions of the Ministry of Education on Deepening Education and Teaching Reform in Universities under the Central Government” and other documents [5, 6]. Based on the relevant documents of the Ministry of Education, major medical colleges and universities have actively promoted the reform of education and teaching, and the quality of talent training has been greatly improved. However, internship teaching is still the weakest link in the stage of medical undergraduate education. “Abandoning internships for postgraduate entrance examinations” and other issues are common [7, 8].

After medical interns enter a hospital for internship, they encounter a different environment in contrast to their school environment; the change from students to semiprofessionals, the change of social environment, and new needs in life and study are generated. Related domestic articles have also put forward many research studies on the needs of college students' Maslow's hierarchy of needs, also known as “the basic hierarchy of needs” by the famous American psychologist Abraham Maslow, 1943; “theory of human motivation” is first proposed in the text, which is divided into physiological needs, security needs, social needs, esteem needs, and self-realization needs in five categories, arranged in order from the lower level to the higher level [9, 10].

In this research, Maslow's need-level theory is applied to the practical teaching work of medical students. Through the results of the questionnaire, in the evaluation of the teaching mode, the overall evaluation of the students in the experimental group is better, and there are significant statistical differences compared with the control group.

The main advantages of students of this teaching model are as follows: they are familiarized in departments and hospitals, rather than just being audiences in schools; teachers' concern is not only about learning but also about life, psychology, and interpersonal relationships. Career planning and many other aspects will be taken care of; and more involved in learning and have a better grasp of knowledge and skills. Through the student's assessment results, it is indeed found that this teaching mode has indeed greatly improved the students' knowledge and skills mastery and has played a real effect of teaching.

Through the questionnaire survey, it is found that by incorporating Maslow's hierarchy of needs theory, the previous notion that students are only for learning knowledge is gradually transformed into students who regard schools as a place to live, study, and develop as a whole, and teachers are also changing this way, in better preaching and receiving karma [11]. Of course, in order to better transform Maslow's level of theory into practical actions in teaching, it is necessary to repeatedly practice certification corrections to form a set of scientific, operability, and beneficial teaching models.

In the current real clinical work, the integration of medical care has become important. Through the integration of medical care, doctors can better obtain the implementation status and feedback of the diagnosis and treatment plans they have formulated, and nurses can better determine the focus of nursing work and the focus of patient education and starting from the patient, a whole. The medical care treatment group also allows patients to have a more sense of belonging, and long-term follow-up management is more effective [12]. However, in the traditional practice teaching work, the medical group and the nursing group are completely separated. The medical group mainly learns the diagnosis of various diseases, treatment measures, and various operating skills according to the requirements of the internship, while the nursing group mainly learns nursing-related knowledge and operations. Skill: the students also express through the questionnaire that through this teaching method, the feeling of being strangers in other departments disappeared. Everyone is a partner in learning and living together, helping each other and promoting each other; and learning together, in the past, each other weak links, such as doctor's diagnosis and treatment feedback, patient follow-up, and theoretical knowledge of nursing, can all complement each other and fill up the shortcomings of knowledge [13, 14]. The assessment results also reflect that through such teaching methods, whether it is for theoretical assessment or various skill operations, it is a great improvement. The reason is, as mentioned above, that common learning and work improve student's initiative ability to learn, discover their own shortcomings in time, increase theoretical knowledge, and improve clinical operating skills.

## 3. Case Study Methods and Observational Indicators

### 3.1. Research Population and Methods

This study includes a total of 134 medical interns who are internships in our department from January to December 2020, including 82 interns, 40 males and 42 females, all with bachelor's degree; 52 nurses, which included 18 boys and 34 girls, all with a college degree; and the age distribution is 20–23 years old. Randomly divide them into the control group and the experimental group, each with 67 people. There is no statistical difference between the two groups in the general information such as gender, age, type of intern, and educational background (*P* > 0.05), and they are comparable.

The control group adopted traditional teaching methods for 67 interns in accordance with the teaching plan and implemented conventional internship teaching in accordance with the internship syllabus, mainly including prejob education, environmental personnel introduction, work attitude, basic knowledge, basic skills, and operations. Trainee doctors and trainee nurses follow the routine work arrangements for internships.

In the experimental group's teaching method, the focus is on combining Maslow's need-level theory, and according to the five levels of needs, it is transformed into practical and operable parts and integrated into the teaching process.

The specific methods are as follows: physiology needs: teachers should take the initiative to care about students' life, work, study, and other aspects in work and in private, help them adjust work and study time, guide work points, relieve work pressure, and care about their daily life, diet, and other aspects; safety needs: in the process of prejob training and internship, the teaching teacher must always put safety education on the focus of teaching, especially the sense of hospitality and occupational protection, set an example, require interns to strictly abide by the operating specifications and teach. Familiar with relevant laws and regulations, strengthen the cultivation of medical ethics and medical style through multiform simulation teaching and strengthen the cultivation of doctor-patient communication, so that students can correctly avoid and deal with doctor-patient disputes; love and belonging needs (emotional needs): this theory is applied in teaching to develop interns and lead. The teacher's entrance meeting will help the interns get familiar with the department environment as soon as possible and create learning conditions for them. At the same time, the teaching teacher pulls in the relationship with the interns and also a teacher and a friend understands the students, so that the students can integrate into the atmosphere of the department; always treat the students as members of the department and eliminate the cognition that they are only learning for a period of time, truly integrated into the big family of the department [15–17]; esteem needs: this need is applied when teachers' pay attention to the cultivation of students' self-confidence and independence and “let go without looking” in the internship. Under the premise of ensuring medical safety, fully mastering skills, and communicating well with patients, students can independently operate some of the tasks they have mastered, improve students' hands-on ability, enhance students' enthusiasm and confidence in medical work, and stimulate their medical beliefs. When a mistake occurs in learning or during practice, the teacher must carefully guide, carefully analyze the cause of the error, find out the corrective measures, and assist in the handling of the problem to communicate well, avoid repeating the same problem in the later work; teachers ought not scold students, learn to respect students, and the students also act as one of their work colleagues, enforcing their enthusiasm for work and not reducing their enthusiasm due to a single mistake [18, 19]; self-actualization needs: this need clarifies the characteristics of interns with different academic qualifications, different majors, different levels, and different employment needs, teaching students in accordance with their aptitude; this need helps teachers fully understand the future needs of students and increase their competitiveness subsequently. This can be done by recognizing outstanding interns in each round to enhance their own value expression. In the internship work, the medical and nursing integrated internship arrangements are carried out, and the medical and nurses unified publicity and education when entering the department, common diseases learn together, integrated teaching, strengthen mutual understanding between medical and nurses, and establish a medical and nursing practice collaboration group to communicate with patients under supervision every week to discuss diagnosis and treatment and nursing work experience.

### 3.2. Observation Indicators

Based on the Korotkoff evaluation model, through an anonymous questionnaire survey by the questionnaire star, the two groups evaluated the relevant evaluations of the internship teaching, and each item is evaluated by graded scores [12, 20, 21]. The “very good” and “good” are recorded as excellent, and “general” and “bad” are recorded as “normal.”

After the internship, a theoretical and technical operation assessment will be conducted. The theoretical assessment will have a total score of 100 points. The skills assessment will take a multistation examination, which mainly assesses patients “doctors” consultations (nurses receiving consultations), doctors' physical examinations (nurses' vital signs determination), and diagnosis and treatment (nursing) plan, 25 minutes per station.

### 3.3. Statistics

Use SPSS 22.0 statistical analysis software is for data processing, measurement data (±*S*) using the *t*-test, and count data (%) represented using the chi-square test. *P* < 0.05, it means that the difference is statistically significant.

## 4. Case Analysis and Comparison

### 4.1. Questionnaire Survey Results

Table 1 provides the results of the two groups of questionnaire surveys. Compared with the control group, the experimental group has statistical differences in all aspects (*P* < 0.05).

### 4.2. Assessment Results

Table 2 provides two theoretical assessment results. Compared with the control group, the experimental group had statistical differences in theoretical assessment and skill assessment (*P* < 0.05).  Table 3 provides the skill assessment results.

## 5. Conclusion

Maslow's hierarchy of needs theory has deeply studied human needs and has been widely used in educational practice. “Integration of medical care” is a collaboration model between medical care and nurses with the patient as the center and rapid recovery as the goal. There is a reasonable division of labor, close contact, information exchange, mutual cooperation, complement, and promotion between doctors and nurses. To sum up, in the clinical practice learning process, through the application of Maslow's need-level theory, the integration of medical and nursing teaching work, and the continuous development of future reform work, can conform the trend of medical education in the new era and conform the reform of medical education. It is required to train more excellent and qualified health personnel.

## Figures and Tables

**Table 1:** Questionnaire results (*n*, %).

Project	Excellent (*n*)		Normal (*n*)		Excellence rating (%)		*X* ^2^	*P*
	Test group	Control group	Test group	Control group	Test group	Control group		
Internship satisfaction	48	32	19	35	71.64	47.76	7.941	0.004
Teaching methods	50	38	17	29	74.63	56.72	4.767	0.022
The effects of teaching methods in learning	52	42	15	25	77.61	62.68	3.564	0.044
Knowledge and skills	49	37	18	30	73.13	55.22	4.674	0.023
Teaching method satisfaction	54	39	13	28	80.60	58.21	7.907	0.004

**Table 2:** Theoretical assessment results $\left(\bar{x}\pm s\right)$.

	Fraction $\left(\bar{x}\pm s\right)$	*t*	*P*
Test group	84.64 ± 4.548	6.471	≤ 0.001
Control group	79.49 ± 4.662		

**Table 3:** Skills assessment results $\left(\bar{x}\pm s\right)$.

	Test group	Control group	*t*	*P*
Inquiry (admission)	20.15 ± 1.87	17.73 ± 2.00	7.222	≤ 0.001
Physical examination (vital signs)	20.06 ± 1.55	17.61 ± 1.82	8.354	≤ 0.001
Development of diagnosis and treatment (nursing) plan	21.01 ± 1.51	18.61 ± 1.64	5.144	≤ 0.001

## Data Availability

The data used to support the findings of this study are available from the corresponding author upon request.
